The article "Analysis of Multifactor-Driven Myopia Disease Modules to Guide Personalized Treatment and Drug Development" was retracted in 2023. Reason: concerns about the peer review.

# Analysis of Multifactor-Driven Myopia Disease Modules to Guide Personalized Treatment and Drug Development

**DOI:** 10.1155/2022/5262259

**Published:** 2022-05-09

**Authors:** Shiliang Liu, Fei Li

**Affiliations:** Department of Ophthalmology, Tongji Hospital, Tongji Medical College, Huazhong University of Science and Technology, Wuhan, 430030 Hubei, China

## Abstract

Myopia is recognized as a multifactor, multicascade complex disease. However, people still know little about the pathogenesis of myopia. Therefore, we aim to guide the personalized treatment, drug research, and development of myopia. Here, based on the interaction network of myopia-related genes, this study constructed a multifactor-driven myopia disease module map. We first identified differentially expressed (DE) miRNAs in myopia. Then, we constructed a myopia-related protein interaction network targeted by these DE miRNAs. Further, we clustered the network into modules and identified module-driven factors, including ncRNAs and transcription factors. Especially, miR-16-5p and miR-34b-5p significantly differentially expressed drive the pathogenic module to influence the progression of myopia. At the same time, transcription factors were involved in myopia-related functions and pathways by regulating the expression of genes in modules, such as Ctnnb1, Myc, and Notch1. In addition, we identified 43 genes in modules that played key roles in the development and progression of myopia such as Vamp2, Egfr, and Wasl. Finally, we constructed a comprehensive multifactor-driven myopia pathogenic module landscape and predicted potential drug and drug targets for myopia. In general, our work not only provided candidates for biological experiments which laid the foundation for the in-depth study of myopia but also has a high reference value for the personalized treatment of myopia and drug development.

## 1. Introduction

Myopia, a highly popular public health problem in the world, has already brought people a huge social and economic burden [1, 2]. Various complications such as retinal detachment, choroidal neovascularization, cataracts, glaucoma, and macular atrophy are more likely to permanently deprive the patient of vision [3]. However, myopia is not only ill-different, but also its pathology and etiology are intricate. Both medical science and biology believe that the occurrence and progress of myopia are affected by both environmental and genetic effects. On the one hand, myopia is affected by a variety of environmental factors, including sleep, working hours, outdoor activities, education level, and daylight intensity [4–6]. On the other hand, many experiments have confirmed that myopia is effectively mediated by genetic factors. For example, Wen et al.'s study showed that C-myc protein can regulate retinal cell apoptosis, leading to form deprivation of myopia associated with retinal degeneration [7]. Immunohistochemistry in mouse eyes performed by Tran-Viet et al. confirmed that SCO2 can encode a copper homeostatic protein that has an effect on mitochondrial cytochrome c oxidase activity in vivo, and the imbalance of the protein can lead to photoreceptor defects and scleral walls. The weakened elasticity leads to thinning of the retina, causing myopia [8]. The form deprivation experiment of guinea pigs by Liu and Sun showed that overexpression of MMP-2 in the sclera mediates the IGF-1/STAT3 pathway, which may be an important cause of myopia formation [9]. Moreover, these studies also provide effective strategies for the prevention and treatment of myopia. For example, Tao et al. performed a form-deprived myopic (FDM) treatment of guinea pigs and found that the sclera cAMP level selectively increased, deducing a therapeutic idea of selectively regulating cAMP to control the progression of myopia by controlling scleral collagen synthesis [10]. These efforts have emphasized the important role of the genome and transcriptome in the pathogenesis of myopia, which has inspired us to further explore the genetics of myopia. Studies have shown that retinoic acid (RA) and Tiam1-Rac1 can regulate mitochondrial dysfunction by activating the P38 MAP kinase pathway and promote apoptosis and differentiation in photoreceptors, which leads to diabetic retinopathy [11, 12]. It may be the underlying pathogenesis of myopia.

We first identified myopia-related differentially expressed miRNA and exacted their target genes from miRTarbase. These targets play a key role in the progression of myopia. Second, a protein-protein interaction (PPI) network of these target genes was constructed, and 43 functional modules were identified as pathogenic modules based on the functions and pathways that these modules were involved in. Then, based on the degree of genes in the module, we identified 43 core driving genes such as Egfr and Wasl, all of which were closely related to myopia. In addition, we identified the ncRNAs such as miR-16-5p, miR-34b-5p, and miR-181b-5p and the transcription factors such as Ctnnb1, Myc, and Notch1 as the main driving factors. Finally, based on the pathogenicity modules, core driving genes, and driving factors, we constructed a comparatively complete module map of myopia dysfunction and expounded the pathogenesis of myopia in multiple dimensions. Moreover, based on these pathogenic modules, we documented that adenosine monophosphate, glutamic acid, aflibercept, and other potential drugs have an important therapeutic effect on myopia. In summary, our study analyzed the role of these multifactor-driven pathogenic modules in myopia, which helps biomedical scientists to investigate further and drug biologists to develop myopia drugs.

## 2. Materials and Methods

### 2.1. Data Resources

Two myopia-related miRNA expression profile datasets were downloaded from the NCBI Gene Expression Omnibus (GEO) database. Among them, GSE84220 contained 6 cases of C57BL/6J normal mice and 6 cases of form deprivation myopia, while GSE58124 contained 12 cases of C57BL/6J normal mice and 6 cases of form deprivation myopia [13]. These myopic mice have been deprived of myopia by induction, followed by RNA extraction with normal mice. Finally, microRNA expression profiles and microarray data analysis were performed, and two sets of miRNA expression profile data were obtained.

### 2.2. Differentially Expressed miRNA Screening

On the one hand, Marfan Syndrome is a unique congenital disorder of connective tissue involving tendons, bones, muscles, eyes, and the cardiovascular system that can lead to joint overactivity, contracture, mild skeletal dysplasia, and high myopia [14, 15]. On the other hand, muscle development, especially the thickening of the eye muscles such as the ciliary muscle, may lead to a decrease in its contractility, causing the inherent dysfunction of myopia [16].

First, background correction and normalization are performed using the background correct function of the R language limma package [17–19]. Then, control probes and low-expression probes were filtered using the arrays function quantile normalization. Finally, the lmFit and eBayes functions of the Lima package of the R language were used to identify differentially expressed miRNAs in the two datasets, respectively, using default parameters.

### 2.3. Construction of Myopia-Related Protein Interaction Network

First, the intersection of two differentially expressed miRNA datasets is performed. Second, mouse miRNA-mRNA target information was downloaded in the miRTarBase database [20] for target prediction of differentially intersecting miRNAs. Then, a protein-protein interaction (PPI) network for target genes was constructed using the String database [21], score > 900.

### 2.4. Mining Functional Module and Identification of Pathogenic Modules

First, the PPIs network was imported into Cytoscape [22–24], and the modules were mined using the ClusterONE plug-in [25]. The parameters were all default values. ClusterONE is a clustering algorithm based on cohesiveness-guided search. It can identify dense substructures in PPI networks as protein complexes. In the ClusterONE algorithm, the higher the cohesion score, the more likely the protein in the group is a protein complex. Then, the R language cluster Profiler package [26] is used for function and path enrichment analysis for each module. Finally, one module was identified as a myopia pathogenic module based on the function and pathway that the module participates in.

### 2.5. Exploring Crosstalking Interactions between Modules

First, use python to write a program that synthesizes the mouse protein interaction network in String (score > 900) to generate 1000 random networks with the network size and each node degree in the unchanged network. Then, we obtained the number of interactions between two modules in random networks and real network according to the random network statistics. Finally, we can identify the significantly crosstalk module pairs. Counting the times (*N*) if the number of interactions in random network was greater than the real number between the module pair. When *p* < 0.05 (*p* = *N*/1000), the interactions between per module pair were considered as significant crosstalk.

### 2.6. Identifying the Driving Genes in Modules

According to the interaction relationships of genes in modules, the connectivity of each module gene was calculated using Cytoscape software. Genes with greater connectivity often represent an active regulatory role within the module. Gene with the highest degree in each module was identified as the driving gene for the pathogenic module.

### 2.7. Identification of Transcription Factors and ncRNAs Significantly Regulating Modules

First, the mouse transcription factor and its target information were downloaded from the TRRUST v2 database [27], and 7,057 interaction pairs with 827 transcription factors were obtained. Then, the mouse ncRNA-mRNA (protein) data was downloaded in the RAID 2.0 database [28] (score > 0.5), and 80343 interaction pairs involving 2310 ncRNAs were obtained. Finally, TFs and ncRNAs significantly regulating modules were identified as driving factors. The driving factor refers to the node with at least two interactions with the module, and the number of interactions significant enriched for per module (hypergeometric test, *p* < 0.05).

In addition, the method was used to predict potential drugs for myopia disease. Drugs and their targets' data were downloaded in the DrugBank database [54], a total of 1,978 target pairs involving 2,755 target genes.

## 3. Results

### 3.1. Identified Differentially Expressed miRNAs

Two miRNA expression profiles were screened, and we obtained 331 (Supplementary Figure S1) and 245 (Supplementary Figure S2) differentially expressed (DE) miRNAs, respectively. Comparing the two datasets, we identified 331 DE miRNAs in both two datasets. These DE miRNAs were considered to be related to myopia.

### 3.2. Constructing the PPI Network of Myopia-Related miRNA Targets

MiRNAs play a core role in the regulation of transcriptional expression of genes. Thus, we exacted the target genes of these 331 myopia-related miRNAs for further elucidating the molecular mechanisms of myopia. As a result, we found that 5,829 genes were regulated by myopia-related miRNAs. These genes may be closely related to the occurrence and development of myopia. and constructed a protein-protein interactions (PPIs) network involving 28574 interactions. This PPI network (Figure 1) is the basis of this study and represents the pathogenesis of myopia mediated by DE miRNAs.

### 3.3. Identified Pathogenic Modules Based on Function and Pathway Classification

It is obviously impractical to carry out meticulous research on the entire protein interaction network. In order to further explore the core regulatory mechanisms of the PPI network, we exacted 43 functional modules from the network. These genes in modules are likely to mean a series of protein complexes or functional pathways that regulate a physiological process together. Thus, we further observed the functions and pathways that the module genes were involved in. A total of 9283 biological process entries, 1045 cellular component entries, 1644 molecular function entries, and 866 KEGG pathways were obtained. The results of the function (Figure 2) and pathway (Figure 3) enrichment analysis indicated that these modules are significantly involved in eye development including the development of camera-type eye and retina development in camera-type eyes. In addition, statistical analysis of functions and pathways revealed that up to 13 modules significantly enriched the biological processes of positive regulation of kinase activity, 11 modules enriched the biological processes of positive regulation of protein kinase activity, and 10 modules enriching regulation of MAP kinase activity, which attracted our attention. Protein kinases, especially MAP kinase, play an important role in the regulation of myopia. In addition, there are 11 modules that are significantly involved in the functions of skeletal system development, gland development, and so on. And 10 modules involved in muscle cell proliferation, positive regulation of cell migration and smooth muscle cell proliferation, and PI3K-Akt signaling pathway, suggesting that myopia is closely related to the skeletal system, hormones, and muscle systems. Considering that, we identified these dysfunctional modules as myopic pathogenic modules, which form a functional network (Figure 4).

### 3.4. Identified Core Driving Genes in Modules

Intergenomic regulation has always been complex and varied. Similarly, the relationship between modules is also complex and diverse. Exploring the complex role of modules will help deepen our understanding of the regulated mechanisms of the pathogenesis of myopia. Therefore, we performed crosstalk analysis between modules based on the interactions between modular genes and identified 83 significant crosstalk interactions (Figure 5). The crosstalk may represent the driving role of the modules and jointly regulate the occurrence and development of myopia. We thought that the driving genes in modules are equally important for the pathogenesis of myopia. Thus, based on the degree distribution of the nodes in modules, the most connected gene in each module was considered to be the most active and most significant driver, a total of 43 driving genes (Figure 6). For example, Vamp2 drives the module 27, the connectivity is as high as 72 Egfr which drives the module 19 with connectivity of 68, and Wasl drives the module 37 with 51 connectivity. These driver genes play an important regulatory role in the module, mediating the formation and development of myopia.

### 3.5. Identified Transcription Factors and ncRNAs Regulating the Pathogenesis of Myopia

Myopia is a multifactor and multicascade complex disease, and the pathogenic module of myopia is naturally regulated by many factors. Transcription factors (TFs) and noncoding RNAs (ncRNAs) have been recognized as disease modifying factors. To explore the role of these regulators in the regulation of myopia, we identified transcription factors and ncRNAs which regulated genes in modules. The results (Figure 7) showed that 72 transcription factors had different degrees of regulation of pathogenic modules. For TFs, Ctnnb1 mediates 8 modules, while Myc, Notch1, Stat3, and other TFs mediate 6 modules, affecting the occurrence and development of myopia. For ncRANs, 511 ncRNAs were identified as driving factors that drive the myopic disease module and play an important role in the progression of myopia. Among these ncRNAs, there were 113 DE miRNAs (Figure 7). The differentially upregulated miR-16-5p and miR-34b-5p regulate seven pathogenic modules, respectively, which have an important impact on the pathogenesis of myopia.

### 3.6. Prediction of Potential Drug and Drug Targets for the Myopia Pathogenic Module

The in-depth exploration of the pathogenesis of myopia is helpful for exploring its therapeutic mechanism, and the prediction of potential drugs and their drug targets is an important value of this study. Here, we predicted potential drugs for pathogenic modules based on the drug and its target relationship. The results (Figure 8) show that 209 drugs may have a pharmacological effect on myopathogenic modules. Among them, adenosine monophosphate and glutamic acid have pharmacological effects on three pathogenic modules and may produce more pronounced therapeutic effects. Drugs such as aflibercept and acetylcysteine have therapeutic effects on two dysfunctional modules and have important implications for the control of the progression of myopia.

## 4. Discussion

Myopia is a symptom where the eye falls before the retina after adjustment of the relaxation state, and the collimated light is refracted by the refraction system of the eye. It has many complications and pathogenic factors, leading biomedical scientists to make very slow progress in their research. However, the social pressure and economic loss resulting from it are increasing day by day, and the in-depth exploration cannot be delayed. Hence, we performed the analysis of multifactor-driven myopia disease modules to guide personalized treatment and drug development. First, we identified DE miRNAs in myopia, and constructed a PPIs network for target genes of DE miRNAs. Further, 43 functional modules were exacted from the PPI network. Functional and pathway enrichment results showed that these modules were significantly involved in the eye- and eye development-related biological processes such as camera-type eye development and retina development in camera-type eyes. Notably, 13 modules significantly enriched the positive regulation of kinase activity, and 11 modules significantly enriched the biological processes of positive regulation of protein kinase activity and regulation of MAP kinase activity. In addition, 11 modules were significantly involved in the development of gland, and 10 modules were involved in muscle cell proliferation and smooth muscle cell proliferation. And Hargrave's study also believes that the extraocular muscle dysfunction caused by extraocular muscles will affect the contraction and abduction interactions between the internal and external muscles, so that the tight elastic fibers behind the cornea stretch and cause the eyeballs to elongate. Refractive errors are closely related [29]. Also worthy of our attention is that 11 modules significantly enriched the biology of gland development. A series of studies have shown that myopia is associated with glands such as meibomian glands [30] and hormones including melanin, melatonin, insulin, glucagon, and secretin [31–33]. And 10 modules were significantly involved in the PI3K-Akt signaling pathway, which acts as a signaling pathway for insulin receptors and plays an important role in the regulation of eye growth and vision (hypermetropia and myopia) [34]. Based on these functions and pathways in which the modular genes are involved in, we identified the functional module as a module of myopia.

Subsequently, we explored driving genes in modules and driving factors for these pathogenic modules. First, we identified 43 driving genes. For example, vesicle-associated membrane protein-2 (Vamp2) is associated with exocytosis of lacrimal gland antioxidants and visual stabilization protein 1, which may cause dry eye disease, photoreceptor synapse damage, and various eye diseases such as diabetic retinopathy leading to the occurrence and development of myopia [35–37]. The epidermal growth factor receptor (EGFR) is thought to regulate adhesion dynamics and corneal epithelial homeostasis during eye development [38, 39]. In addition, in previous studies, WASL was found to be differentially expressed in transgenic *β*B1-crystallin-MYOC mice, which may be related to ocular cell adhesion and cell-matrix interactions [40]. All of these driver genes were associated with the eye function, driving the pathogenic module. Then, transcription factors (TFs) and noncoding RNAs (ncRNAs) that are recognized as disease-modifying factors were identified. For example, *β*-catenin (Ctnnb1) plays a key role in cell adhesion, Wnt/*β*-catenin, and Wnt signaling pathways, which are closely related to corneal epithelial delamination and eye development [41, 42]. C-myc protein can regulate retinal cell apoptosis, which leads to retinal degeneration. It is closely related to the progression of myopia [7]. Notch1 plays an important role in epithelial differentiation, which is closely related to the corneal repair and the differentiation of ganglion cells and photoreceptors [43, 44]. MMP-2 overexpression mediated by the IGF-1/STAT3 pathway in the sclera plays a key role in the development of myopia and scleral remodeling [45, 46]. In addition, miR-34 families, miR-16-5p, miR-15b-5p, and other miRNAs play an important mediating role in the pathogenic module and are differentially upregulated in myopia mouse models. Studies by Ye and Steinle have confirmed that the expression of miR-34a increases in the lens and blocks Mitochondrial energy metabolism and enhances cytochrome C release by inhibiting Notch2, which triggers mitochondria-mediated apoptosis and oxidative stress [47]. MiR-15b and miR-16 have been shown to play a role in suppressing insulin resistance by reducing TNF*α* and SOCS3 signaling and increasing IGFBP-3 expression. This protects the retinal endothelial cells (REC) against hyperglycemia-induced apoptosis and has been identified as a potential therapeutic target for the treatment of diabetic retinopathy [48].

Finally, combining with the myopia pathogenic module and its multifactor driving factors, we constructed a comprehensive map of the myopia dysfunction module and predicted the potential drugs and their drug targets. The prediction results showed that drugs such as adenosine monophosphate, glutamic acid, and aflibercept have potential pharmacological effects on the occurrence and development of myopia. These predictions have been widely confirmed and confirmed in previous experiments. For example, studies by Guoping et al. confirmed that cyclic adenosine monophosphate activates retinal apolipoprotein A1 expression and inhibits myopia growth [49]. Ikuno et al.'s study showed that glutamic acid can regulate excitatory neurotransmitters in the retina and thus play a pivotal role in eye development and lens-induced myopia (LIM) [50]. Several studies have shown that aflibercept has long been used to promote the formation of choroidal neovascularization in myopia [51–53]. Therefore, previous studies have demonstrated the validity of our results.

## 5. Conclusion

In summary, we have obtained a more complete myopia disease module map. This map provides a number of proven myopia-driven genes and candidate molecules to be tested, providing a theoretical basis for the further study of myopia. In addition, based on this map, we have predicted a series of potential drugs that may serve as important targets for drug retargeting by drug developers. However, there are still several limitations in our study. We need to do more experiments and get a general conclusion. Our finding grounds the future study of myopia and provides a significant reference for personalized treatment of myopia and drug development.

## Figures and Tables

**Figure 1:** Target protein interaction network.

**Figure 2:** GO enrichment analysis.

**Figure 3:** KEGG pathway enrichment analysis.

**Figure 4:** Module function network.

**Figure 5:** Crosstalk relationship between modules.

**Figure 6:** Degree of interaction within the module.

**Figure 7:** TF and ncRNA pivot analysis.

**Figure 8:** Comprehensive map of multiple factors driven myopia pathogenic modules.

## Data Availability

The datasets used and/or analyzed during the current study are available from the corresponding author on reasonable request.

## Supplementary Materials

Supplementary Materials Two miRNA expression profiles were screened, and we obtained 331 (Supplementary Figure S1) and 245 (Supplementary Figure S2) differentially expressed (DE) miRNAs, respectively.
